# Steeling Ourselves: Intragroup Communication while Anticipating Intergroup Contact Evokes Defensive Intergroup Perceptions

**DOI:** 10.1371/journal.pone.0131049

**Published:** 2015-06-22

**Authors:** Hedy Greijdanus, Tom Postmes, Ernestine H. Gordijn, Martijn van Zomeren

**Affiliations:** Department of Social Psychology, University of Groningen, Groningen, The Netherlands; University of New South Wales, AUSTRALIA

## Abstract

Two experiments investigated the role of intragroup communication in intergroup conflict (de-)escalation. Experiment 1 examined the effects of intragroup communication (vs. individual thought) and anticipated face-to-face intergroup contact (vs. no anticipated face-to-face intergroup contact). The group discussions of stigmatized group members who anticipated face-to-face intergroup contact revolved more around intergroup hostility. This boosted ingroup identification and increased social creativity but also led to steeling (a hardening of perceived intergroup relations). In Experiment 2, new participants listened to the taped group discussions. The discussions of groups anticipating face-to-face intergroup contact evoked more intergroup anxiety-related discomfort than discussions of groups not anticipating face-to-face intergroup encounters. Together, these results support the idea that steeling is a defensive reaction to prepare for an anxiety-arousing intergroup confrontation. Although steeling is also associated with positive consequences such as increased ingroup solidarity and social creativity, this hardened stance may be an obstacle to conflict de-escalation.

## Introduction

Although the term *intergroup conflict* instills the image of a clash between groups, paradoxically conflict flourishes when there is a lack of contact and groups do *not* interact [1]. We propose that *intra*group processes can help explain this phenomenon. Intragroup communication can shape intergroup perceptions, and may therefore be essential in conflict (de)escalation. Specifically, the current research investigated how intergroup perceptions evolved in small groups that talked among each other about an anticipated face-to-face intergroup contact situation. In conflict situations where the outgroup holds negative views about the ingroup, such anticipation of contact may be threatening. We hypothesized that intragroup discussion may cause shared construal of anticipated contact as hostile but simultaneously offers members of stigmatized groups an opportunity to steel themselves in anticipation. We conceptualize steeling as a state of psychological preparation for a stand-off with an outgroup holding negative views of the ingroup. We will argue that in such situations steeling can consist of defensive “upgrading” of ingroup perceptions, downgrading of outgroup perceptions, or both.

### Anticipating Intergroup Contact

When and how intergroup contact reduces prejudice have been focal questions for the field of intergroup relations research at least since Allport [2], if not before (see [3] for a review). Meta-analyses have demonstrated that positive contact typically reduces intergroup prejudice [3]. But it has also been noted that, in practice, positive contact between conflicting groups may be quite uncommon due to self-segregation [4]. One reason for this may be that intergroup contact can be threatening [5] particularly for stigmatized groups. Because expectations of problematic contact motivate avoidance of intergroup contact [6–8] interventions may involve organizing intergroup encounters. But what happens in the run-up to these arranged meetings? Specifically, how do stigmatized group members *prepare* for an upcoming intergroup encounter?

Even though actual intergroup contact may be quite rare, it appears that thoughts that prepare individuals for how to behave in contact situations are readily activated. Indeed, priming with an outgroup activates not just stereotypes, but also concepts associated with the relationship that one entertains with that group (e.g., priming with gay men activates hostile behavior and priming with doctors activates patient behavior—also depending on participants’ implicit attitudes [9,10]). The expectations and motivations with which group members approach intergroup contact are important factors in whether contact facilitates conflict de-escalation or escalation [11]. When people anticipate interacting with a potentially antagonistic outgroup, various processes take effect. First, individuals are concerned with how outgroup members perceive them: Meta-stereotypes of how “they” think about “us” are activated [12,13]. When these meta-stereotypes are negative, this can be threatening (i.e., evoke intergroup anxiety [5]), intensify negative intergroup perceptions [14] and foster self-defensive responses [15]. Principally, if leaving such a stigmatized group is impossible or not desired group members may feel the urge to affirm or establish a positive feeling about the ingroup by upgrading perceptions of the ingroup, downgrading perceptions of the outgroup, or a combination of both. For example among other consequences, anticipated or actual devaluation may increase ingroup identification [15], outgroup derogation [16], and *social creativity*–the re-valuation of negative traits attributed to the ingroup as positive (e.g., *Black is beautiful*[17,18]). In both these processes of upgrading perceptions of the ingroup and of downgrading perceptions of the outgroup, we propose that intragroup communication plays a central role.

### The Role of Communication

Humans spend most of their time within their own ingroups [19]. And through communication in such fairly homogeneous intragroup settings, our understanding of reality (particularly social reality) is shaped [20–23]. This process is particularly important for understandings of “us” and “them,” which mainly acquire meaning through intragroup communication [24]. Through intragroup interactions, we piece together who we are and what we do [23,25] but also who “they” are, how they see us, and what we should do about them [26,27] (e.g., Smith & Postmes, 2009, 2011). Thus group members actively construct and adjust a sense of shared social identity and consequent perceptions, norms, and attitudes [28–30].

Research on *extended* intergroup contact [31] illustrates the importance of this process. Through other ingroup members, people may learn about positive contact between ingroup and outgroup members. Such extended contact improves intergroup relations [32–34]. Multiple processes are involved: Extended contact lowers intergroup anxiety, but it also fosters positive norms concerning contact [35]. It appears, then, that learning about others’ positive encounters with an outgroup member does not merely inform one’s perceptions of “them”, but also helps shape group norms about how to behave towards “them” (cf. [36–38]).

However, when people anticipate having contact with potentially stigmatizing outgroups, one might hypothesize that they are not so likely to share positive stories but rather discuss past and future negative encounters. Studies of imagined intergroup contact indeed suggest that intergroup anxiety hinders the ability to imagine positive contact [39] (see also [40]). This may be because intragroup communication typically emphasizes information that is consistent with shared perceptions [41,42] (see also [43]). Anticipated intergroup contact may thus facilitate discussion of negative intergroup encounters if the anticipations are negative. Additionally, there may be a motivational component: Anticipated intergroup contact may be biased towards information that fosters coalition building *against* a conflicting outgroup [44]. In sum, for various reason intragroup communication is more likely to dwell on personal anecdotes of intergroup hostility—and such anxiety-related information likely influences group members’ cognition more than anxiety-unrelated information [45].

Once discussions involve negative examples of intergroup contact, for instance taking the form of anecdotes describing personal experiences with intergroup hostility, this may increase the vividness of the threat posed by the outgroup, affecting group members’ perceptions and promoting defensiveness (cf. [46–48]). Importantly, communication acts as a double-edged sword—not only shaping what receivers of communication think but also what senders of communication think. People generally come to believe the things they say [49–51] and forget information that is not discussed by themselves (cf. retrieval-induced forgetting [52]) or their communication partners [53] (for reviews see [54,55]). Accordingly, perceptions of the intergroup relationship may become more negative after sharing hostility anecdotes. But simultaneously, it is likely that the confrontation with others’ negative stigmatizations will result in a positive reappraisal of the supposedly negative ingroup traits (i.e., a process of social creativity). This dual process of hardening attitudes towards “them” whilst boosting pride in “us” is what we refer to as *steeling* in this paper.

For this process of steeling to take effect, we expect that the anticipation of actual face-to-face intergroup contact plays a crucial role in determining whether such intergroup hostility anecdotes are indeed discussed or not. This is because anticipated face-to-face contact, especially between groups in conflict, is crucial to raise the threat levels and concerns that invoke these interactive group processes. In line with a conception of individuals’ cognition as emergent in social contexts [56,57], it has often been argued and shown that the intergroup context in which intragroup interactions take place is one important factor that determines the directions in which perceptions develop [58–61]. Thus, in the current research we hypothesized that steeling is particularly likely when intergroup contact is anticipated and group members are provided with an opportunity to discuss the outgroup among themselves.

### Current Research

What are the conditions in which communication becomes an important factor in this process of steeling (in addition to the other processes already mentioned above, e.g., [15,16])? Communication will likely exert less influence when intergroup relations have become entrenched, for example through socialization. Conversely, communication may exert greater impact when group members have something meaningful to share about the intergroup situation—in artificial groups, social sharing might therefore be less important than in existing groups (cf. [62,63]). By using pre-existing groups in a real conflict and targeting fairly new members who have engaged in relatively little intragroup communication and socialization about this conflict, the current experiments sought to create an optimal environment to examine the influence of intragroup communication on steeling against intergroup hostility.

We examined effects of unconstrained intragroup communication in small groups (versus individual thought) and anticipated face-to-face intergroup contact (versus no anticipated face-to-face contact) on steeling. In this research, we invited real group members, engaged in a genuine intergroup conflict, into the laboratory. Linking research on intergroup conflict with shared reality and social identity, we hypothesized that intragroup communication while anticipating intergroup contact leads to activation of negative meta-stereotypes (rather than stereotypes) as group members construe contact as hostile and, consequentially, this communication results in steeling.

#### Intergroup conflict characteristics

In order to understand the nature of the experiments below, it is necessary to provide some background detail to the intergroup conflict which we examined. We focused on an actual conflict between students in Groningen and their outgroup *“stadjers*,*”* which is similar to the town-gown distinction that is common to many University cities. In Groningen, *stadjers* is a non-evaluative term for non-student city inhabitants that is also used by formal authorities. Stadjers stereotype students as intelligent and sociable, yet noisy litterers. This intergroup distinction is relevant to students for several reasons. For instance, many streets in Groningen have a student inhabitant quotum and students have to find new housing if they are too many. The idea has also been voiced to relocate all students outside the city to reduce disorder and conflict. So for students the conflict is characterized by negative meta-stereotypes and social stigmatization of the ingroup as troublesome outsiders. They are stigmatized in the very real sense of possessing “a social identity that is devalued in a particular social context” [64] (p. 505): Stadjers do not want them as their neighbors.

The reverse stereotype that students have about stadjers mostly appears to reflect the irritations that students cause (e.g., old-fashioned nags). It is also worth noting that the conflict between the groups may cause students to experience discomfort around stadjers but is unlikely to arouse strong feelings of (physical) threat (even though there are regular reports of violence against students which may be classified as intergroup violence). A student anticipating intergroup contact will probably expect to meet with prejudice and verbal hostility rather than aggression or violence.

#### Operationalizations of steeling

We expected steeling to manifest itself in specific ways. As mentioned, steeling can consist of defensive “upgrading” of ingroup perceptions, downgrading of outgroup perceptions, or both. Although these effects can manifest in several ways, we focus on three measures of steeling.

First, students can enhance the *relative* positivity of the ingroup by reciprocating group-level negativity (cf. [65]). Our prediction was that students would raise more negative thoughts about the outgroup when communicating in a group whilst anticipating intergroup contact. Accordingly, participants should report more negative collective attitudes of the ingroup towards the outgroup—*we* do not like *them*. Thus, in the current conflict—which is dominated by an outgroup holding negative views of the ingroup rather than the reverse—we expected group members to counteract the negativity imbalance by expressing that the ingroup holds negative views of the outgroup as well. This is the first manifestation of steeling we focus on.

A second way in which steeling could manifest is social creativity [18]. We operationalized social creativity by examining the valuation of *meta-stereotypes*–the valuation of the traits by which the outgroup stigmatizes the ingroup (cf. [66]). Such stigmata are often intended negatively, but during intragroup communication they can be reappropriated and romanticized (cf. identity performance [67]). Thus, the second measure of steeling we included is that meta-stereotypes should become more positively valenced (or romanticized).

The third measure of steeling in the current research is ingroup identification. Prior research has shown that ingroup devaluation may increase ingroup identification [15] (see also [68]). Accordingly, we expected that participants who anticipated face-to-face intergroup contact to report increased ingroup identification after intragroup communication.

#### Control Measures

The function of steeling is the bolstering of the ingroup in preparation for a potential stand-off when contact is anticipated. Thus, steeling focuses primarily on “us”, not on “them”. Accordingly, perceptions of what exactly the outgroup thinks and does should not be affected by steeling. We added four control measures to verify this.

As a first control measure, we gauged perceptions of the outgroup’s attitude towards the ingroup—which were presumably negative in the current conflict. Downplaying this source of anxiety is difficult because the threat may be hard to deny (cf. [69])–and if group members do manage to laugh away any suggestion of threat (as in groupthink [70]), this may severely hamper their preparation for a subsequent hostile confrontation. Two additional control measures concerned participants’ valence judgments of stereotypic traits and their application of stereotypes to the outgroup. Finally, meta-stereotype application was included as a control measure to verify that students romanticize meta-stereotypes (i.e., social creativity) without simultaneously perceiving stadjers as having a more positive attitude towards them (cf. the outgroup’s attitude towards the ingroup as a control measure) or as applying fewer meta-stereotypes. These latter effects would not be effective steeling because overly positive expectations intensify negative affective reactions during the actual intergroup encounter rather than buffer against anticipated hostility.

### Summary

To sum up, we hypothesized that intragroup communication while anticipating intergroup contact 1) leads group members to discuss personal experiences with ingroup-directed hostility and 2) activates negative meta-stereotypes, both of which consequentially result in 3) steeling against anticipated hostility. This steeling should manifest itself in 3a) more negative collective perceptions of the outgroup, 3b) more positive perceptions of meta-stereotypes, and 3c) increased ingroup identification. We also included various control measures on which we did not expect effects of anticipated contact (see below).

As mentioned, the intragroup communication resulting in steeling should create a shared reality of the anticipated face-to-face intergroup contact as hostile and uncomfortable, and activate negative meta-stereotypes. Communication content (i.e., presence of intergroup hostility anecdotes) and meta-stereotype activation should thus mediate the steeling effects. This is tested in Experiment 1. Furthermore, a follow-up Experiment 2 tested the impact of the taped discussions on listeners. We expected that listening to groups anticipating face-to-face intergroup contact would evoke more discomfort in a separate sample of participants belonging to the same ingroup than listening to ingroup members discussing the outgroup without anticipating direct intergroup contact.

## Experiment 1

### Method

#### Ethics statement

This research was approved by the Ethical Committee Psychology of the University of Groningen (approval numbers: 09142-N, 10113-N, ppo-011-216). All participants provided their written informed consent. Questionnaire data of Experiments 1 and 2 are available in supplemental files S1 Dataset and S2 Dataset, respectively. We report all details of both experiments (all included and excluded participants, conditions, and variables).

#### Participants and design

One hundred and thirty-four students (51 men, age *M* = 19.87, *SD* = 2.28) were randomly assigned to a 2 (no anticipated face-to-face contact, anticipated face-to-face intergroup contact) X 2 (individual thought, intragroup communication) between-subjects design. For ease of interpretation, this design collapses three conditions lacking anticipated face-to-face contact. In the original (full) design, anticipated face-to-face intergroup contact was compared with: a) no intergroup contact, b) one-way written communication (sending the outgroup a message), or c) two-way written communication (sending a message and receiving one back). These conditions were designed to test whether anticipating intergroup communication in itself would have any effects (independently of anticipated *face-to-face* contact). Helmert contrasts indicated no differences between any of the control conditions (a-c) on any of the measures reported, *p*s > .10. We thus simplified the design by collapsing the controls, statistically correcting for the different *n*s. To correct for the different sample sizes per condition, corrected contrasts were computed for each of the four conditions as: Original contrast * (*N*_total_ / (*N*_condition_ * number of conditions)). Important to note is that analyses of the full 4X2 design, as well as analyses uncorrected for sample size, generated similar patterns of results.

#### Procedure

The communication manipulation was similar to that of Smith and Postmes (2011). After giving informed consent, participants received written instructions to “form an impression of the intergroup situation,” through either a 5-minute discussion with students (*intragroup communication* condition) or individual paper-and-pencil thought-listing (*individual thought* condition).

In the *anticipated face-to-face contact* condition, participants formed this impression to prepare for a real-life intergroup discussion (of which no further details were provided). In the *no anticipation* control condition, they formed this impression without reference to face-to-face intergroup discussion. Subsequently, they individually filled out paper-and-pencil questionnaires including the focal dependent variables and some exploratory measures. The exploratory measures gauged participants’ impressions of the intergroup situation (open-ended), perceived intergroup conflict, ingroup-outgroup overlap, inter- and intragroup distinctiveness, familiarity with and stereotypicality of discussion partners, consensualisation and validation of (meta-)stereotypes, and personal opinions on intergroup contact-related issues. Because these measures were exploratory, the current paper focuses on the steeling measures but details are available upon request. All participants started with a (meta-)stereotype activation questionnaire, then filled out questionnaires measuring steeling and control variables ending with a questionnaire on (meta-)stereotype valence, open-ended questions on participants’ thoughts on the research questions and hypotheses, and demographic questions. Finally, participants were debriefed. Audio recordings of the intragroup discussions were transcribed for analysis.

#### Measures

To measure hostility anecdotes, transcribed discussions were coded separately by the first author and a coder blind to the hypotheses and conditions. They coded whether (mild) intergroup hostility was mentioned (*hostility anecdotes*; 1 = someone reported a personal experience with hostile outgroup members, 0 = no-one did this). We chose this 0/1 coding scheme rather than counting anecdotes within discussions because typically one participant shared a hostility anecdote, eliciting sympathizing reactions by others. One example from the anticipated face-to-face contact condition was: “I always have quarrels with my upstairs neighbors about noise by day.” A participant in the no anticipation condition told: “The other day, there was hassle about parked bikes. It’s usually about that. It’s about bikes or about noise.” Because the presence or absence of such hostility anecdotes was rather straightforward coders were in 100% agreement and, hence, reliability statistics could not be computed.

The (meta-)stereotype activation questionnaire consisted of 28 incomplete words. Instructions were: “Below you see some incomplete words. Replace all dashes with one letter to create existing words. Provide the first correct solutions that come to mind.”–followed by an example and all items. Fourteen could be completed to stereotypes, another 14 to meta-stereotypes. All stimuli could also be completed to words not associated with the current intergroup context (e.g., *_ _ _ _ ruchtig* could be completed to *luidruchtig* [meta-stereotype: noisy], or *roemruchtig* [illustrious]). We obtained (meta-)stereotypes from a pilot study (*N* = 104) in which students answered the open-ended questions “What do students think stadjers in general think of them?” and “What do students in general think of stadjers?”. The most frequently mentioned (> 20%) meta-stereotypes (noisy, arrogant, stuck up, social, partying, clever, lazy) and stereotypes (kind, lumpish, rigid, rough, nagging, old-fashioned, stupid) and synonyms (e.g., *intelligent*, *friendly*) were randomly interchanged in one questionnaire, and (meta-)stereotype activation was measured as the total number of words completed to (meta-)stereotypic traits (cf. [71,72]). These word completion targets were not balanced for word frequency.

We operationalized steeling with the measures *ingroup’s attitude towards the outgroup*, *meta-stereotype valence*, and *ingroup identification*.

The ingroup’s attitude towards the outgroup concerned individual group members’ perceptions of this attitude as measured with the question “How positive or negative do you think students in general view stadjers?” on a scale from -3 (*negative*) to 3 (*positive*).

Meta-stereotype valence was measured using scales gauging participants’ individual evaluation of (meta-)stereotypes from -3 (*negative*) to 3 (*positive*). Meta-stereotype valence thus measured participants *personal* evaluations of these traits, which may vary regardless how they think the outgroup evaluates these traits (i.e., independently of the outgroup’s attitude towards the ingroup).

Identification was measured using a multi-component measure (Leach et al., 2008; overall Cronbach’s α = .90) on a 7-point scale. Because effects on each component were broadly similar, we only report the aggregate score.

As mentioned above, at least in the current intergroup conflict steeling is an ingroup-centered process and accordingly perceptions of the outgroup need not be affected by it. Therefore, we added four control measures on which we did not expect effects: the *outgroup’s attitude towards the ingroup*, *stereotype valence*, *stereotype application*, and *meta-stereotype application*.

The outgroup’s attitude towards the ingroup and stereotype valence were measured similar to the steeling measures of, respectively, the ingroup’s attitude towards the outgroup and meta-stereotype valence.

Stereotype application was measured with seven stereotypes (e.g., “Old-fashioned: To what extent do *you* think this characteristic applies to the outgroup?” 1 *absolutely not* to 7 *absolutely)*, randomly interchanged with seven meta-stereotypes as fillers. The meta-stereotype application comprised seven meta-stereotypes (e.g., “Noisy: To what extent do you think the *outgroup* applies this characteristic to students?”) and seven stereotypes as fillers. Correlations between the steeling and control measures are depicted in Table 1.

**Table 1:** Correlation Matrix of Steeling and Control Measures.

	1.	2.	3.	4.	5.	6.	7.
Steeling measures							
1. IG’s attitude towards OG	1.00						
2. Meta-stereotype valence	-0.09	1.00					
3. Ingroup identification	-0.11	0.44**	1.00				
Control measures							
4. OG’s attitude towards IG	0.25**	-0.01	-0.07	1.00			
5. Stereotype valence	0.12	0.27**	-0.14	0.14	1.00		
6. Stereotype application	-0.35**	0.05	0.18*	-0.35**	-0.10	1.00	
7. Meta-stereotype application	-0.13	0.04	0.22*	-0.30**	-0.15	0.55**	1.00

*Note*: IG = ingroup, OG = outgroup.

* Pearson’s correlation *p* ≤ .05.

** Pearson’s correlation *p* ≤ .01.

### Results

The open-ended questions about research questions and hypotheses revealed that participants were unaware of the expected results. Within-condition Mahalanobis distance analyses revealed no outliers.

#### Analytic strategy

Because participants were nested within discussion groups with intraclass correlations in communication conditions ranging from .002 (for meta-stereotype valence) to .317 (for meta-stereotype application), data were analyzed with multilevel regressions in HLM (Raudenbush, Bryk, & Congdon, 2004). One-tailed, Bonferroni-corrected tests generated similar results as the conservative two-tailed tests reported here. For comparing intragroup communication and individual thought, participants in the individual thought condition were divided into nominal groups (i.e., participants went through the procedure described earlier individually, but data were clustered within randomly assigned groups for multilevel analyses). This procedure resulted in a final sample of 27 groups of two to three students in this condition, equal to the intragroup communication condition.

We expected one cell mean (i.e., intragroup communication while anticipating intergroup contact) to differ from the others. In such a non-crossover interaction, omnibus *F*-tests may erroneously suggest absence of the hypothesized pattern [73]. Therefore we used hypothesis-specific, planned contrasts [74] (cf. [75,76]). To test the hypothesis that intragroup communication while anticipating intergroup contact would instigate steeling, this condition was compared with the remaining conditions using a Helmert contrast (contrast1). There were two control contrasts to investigate two alternative hypotheses. To test for the influence of individual thought while anticipating intergroup contact on steeling, this condition was compared with both intragroup communication and individual thought without anticipated face-to-face contact (contrast2). A third contrast compared steeling after intragroup communication without anticipated face-to-face contact with steeling after individual thought without anticipated face-to-face contact (contrast3).

The estimated HLM models for the (meta-)stereotype activation, steeling, and control measures were:

$$\text{Level-1: }Y=\;\beta_{0}+r$$

$$\text{Level-2: }\beta_{0}=\;\gamma_{00}+\;\gamma_{01}*\;\left(\text{contrast1}\right)\;+\;\gamma_{02}*\;\left(\text{contrast2}\right)\;+\;\gamma_{03}*\;\left(\text{contrast}3\right)\;+u_{0}$$

*Y* represents the dependent variable (i.e., one of the steeling or control measures), β is the individual-level regression coefficient, γs are group-level regression coefficients, and *r* and *u* respectively are the individual-level and group-level errors.

We conducted multilevel analyses to test for effects of hostility anecdotes on steeling and control measures. A dummy variable (hostility anecdotes) indicated whether or not groups shared hostility anecdotes.^7^

The estimated HLM models were:

$$\text{Level-1: }Y=\;\beta_{0}+r$$

$$\text{Level-2: }\beta_{0}=\;\gamma_{00}+\;\gamma_{01}*\;\left(\text{hostility anecdotes}\right)\;+u_{0}$$

Again, *Y* represents the dependent variable, β the individual-level regression coefficient, γs group-level regression coefficients, and *r* and *u* respectively the individual-level and group-level errors.

#### Intragroup communication content

Because there was no communication content to analyze in the individual thought conditions, all analyses in this subsection concern the intragroup communication conditions. One discussion was not recorded, hence the final sample consisted of 26 discussions. Group-level Pearson’s *χ* ^2^-test revealed that 83% of groups anticipating intergroup contact shared hostility anecdotes, compared to 30% of control groups, *χ* ^2^ (1) = 5.38, *p* = .02.

Results of multilevel analyses indicated that in those groups where hostility anecdotes were shared, group members perceived their ingroup’s attitude towards the outgroup more negatively, *t*(24) = -2.14, *p* = .04, romanticized meta-stereotypes more, *t*(24) = 1.89, *p* = .07, and identified more strongly with their ingroup, *t*(24) = 3.04, *p* < .01, than in the other groups. There were again no significant influences on the complementary control measures outgroup’s attitude towards the ingroup and stereotype valence, *p*s > .69. Analyses with *hostility anecdotes* as predictor were statistically corrected for the different numbers of groups that did or did not communicate about these experiences (cf. Footnote 2). Uncorrected analyses generated similar results.

#### Activation of (meta-)stereotypes

There were no significant effects on meta-stereotype or stereotype activation, *p*s > .20, possibly due to differences in word frequency between (meta-)stereotypic and unrelated solutions. On average, participants completed 5.97 stimuli to meta-stereotypes (*SD* = 1.95) and 5.06 to stereotypes (*SD* = 2.11). Because there was no effect on meta-stereotype activation, we did not test its hypothesized mediating role in steeling.

#### Steeling

For an overview of within-condition means and standard errors of all steeling and control measures, see Table 2.

**Table 2:** Means and Standard Errors (in Brackets) for Steeling and Control Measures.

	No face-to-face intergroup contact anticipation		Anticipated face-to-face intergroup contact	
	Individual thought	Intragroup communication	Individual thought	Intragroup communication
Steeling measures				
IG’s attitude towards OG	0.39 (0.38)	0.14 (0.38)	0.62 (0.47)	-1.00 (0.34)***
*scale range* ^-^ *3–3*				
Meta-stereotype valence	-0.10 (0.15)	-0.08 (.15)	-0.05 (.19)	0.34 (0.14)**
*scale range* ^-^ *3–3*				
Ingroup identification	4.92 (0.23)	4.93 (0.23)	4.73 (0.28)	5.36 (0.20)*
*scale range 1–7*				
Control measures				
OG’s attitude towards IG	-1.17 (0.34)	-0.79 (0.34)	-0.68 (0.42)	-1.27 (0.30)
*scale range* ^-^ *3–3*				
Stereotype valence	-0.82 (0.17)	-0.84 (0.17)	-0.80 (0.20)	-0.99 (0.15)
*scale range* ^-^ *3–3*				
Stereotype application	3.85 (0.24)	4.21 (0.24)*	4.35 (0.30)	4.70 (0.21)**
*scale range 1–7*				
Meta-stereotype application	5.32 (0.20)	5.38 (0.19)	5.41 (0.24)	5.57 (0.17)
*scale range 1–7*				

*Note*: IG = ingroup, OG = outgroup.

* Helmert contrast comparing this condition to all conditions to the left *p* ≤ .05.

** Helmert contrast comparing this condition to all conditions to the left *p* ≤ .01.

*** Helmert contrast comparing this condition to all conditions to the left *p* ≤ .001.

Fig 1 shows the effects on the ingroup’s attitude towards the outgroup. Results support the hypothesis that when intergroup contact is anticipated, the opportunity for intergroup communication leads to more negative perceptions, compared with the other conditions, γ = -1.05 (*SD* = 1.86), *t*(50) = -3.66, *p* = .001. This γ coefficient means that, controlling for the effects of the other contrasts and the multilevel structure of the data, participants who engaged in intragroup communication while anticipating intergroup contact perceived their ingroup’s attitude towards the outgroup, on average, 1.05 points lower on a 7-point scale than participants in the remaining three conditions. As expected, the control contrasts were non-significant, *p*s > .34. In line with the nature of the current intergroup conflict, participants’ average rating of the ingroup’s attitude towards the outgroup *overall* did not significantly differ from zero (i.e., neither positive nor negative), overall intercept = 0.17, *t*(53) = 1.33, *p* = .19.

**Fig 1:** Effects of intragroup communication and anticipated face-to-face intergroup contact on ingroup’s attitude towards the outgroup. Error bars represent 95% confidence intervals, scale ranged from -3 (*negative*) to 3 (*positive*). Intragroup communication while anticipating face-to-face intergroup contact (contrasted to the other three conditions) leads to more negative perceptions of the ingroup’s attitude towards the outgroup.

Fig 2 shows the effects on meta-stereotype valence. Hypothesis tests indicated, in line with expectations, that intragroup communication while anticipating intergroup contact yielded more positive evaluations of meta-stereotypes, γ = 0.34 (*SD* = 1.33), *t*(50) = 2.96, *p* < .01. This γ coefficient means that, controlling for the effects of the other contrasts and the multilevel structure of the data, participants who engaged in intragroup communication while anticipating intergroup contact rated meta-stereotypic traits, on average, 0.34 points higher on a 7-point scale than participants in the remaining three conditions. As expected, the control contrasts were non-significant, *p*s > .35. Split analyses revealed that communication while anticipating intergroup contact yielded more positive evaluations of positive meta-stereotypes, *t*(50) = 2.32, *p* = .02, and less negative evaluations of negative meta-stereotypes, *t*(50) = 2.96, *p* < .01. Control contrasts were non-significant, *p*s > .25. On average, meta-stereotype valence did not differ from zero (*M* = -0.04), *t*(53) = -0.75, *p* = .46.

**Fig 2:** The effects of intragroup communication and anticipated face-to-face intergroup contact on meta-stereotype valence. Error bars represent 95% confidence intervals, scale ranged from -3 (*negative*) to 3 (*positive*). Intragroup communication while anticipating face-to-face intergroup contact (contrasted to the other three conditions) leads to romanticization of meta-stereotypic traits.

Fig 3 shows the effects on identification. In line with expectations, intragroup communication while anticipating intergroup contact led participants to identify more strongly with their ingroup, γ = 0.37 (*SD* = 1.94), *t*(50) = 2.19, *p* = .03. This γ coefficient means that, controlling for the effects of the other contrasts and the multilevel structure of the data, participants who engaged in intragroup communication while anticipating intergroup contact rated their ingroup identification, on average, 0.37 points higher on a 7-point scale than participants in the remaining three conditions. As expected, the control contrasts were non-significant, *p*s > .56. Participants’ average ingroup identification was above-midpoint (overall intercept 4.95, *t*(53) = 21.93, *p <* .001).

**Fig 3:** The effects of intragroup communication and anticipated face-to-face intergroup contact on identification. Error bars represent 95% confidence intervals, scale ranged from 1 to 7. Intragroup communication while anticipating face-to-face intergroup contact (contrasted to the other three conditions) increases group members’ identification with their ingroup.

#### Control measures

Consistent with the nature of the current intergroup conflict, participants perceived negative attitudes of the outgroup towards their ingroup (overall intercept -0.98), *t*(53) = -9.55, *p* < .001. As expected, none of the contrasts affected this control measure, *p*s > .10. As hypothesized, none of the contrasts affected stereotype valence, *p*s > .43. On average, participants valued stereotypes negatively (overall intercept -0.84), *t*(53) = -17.42, *p* < .001. Intragroup communication while anticipating intergroup contact unexpectedly led participants to apply more stereotypes to the outgroup, γ = 0.50 (*SD* = 2.08), *t*(50) = 2.77, *p* < .01. This γ coefficient means that, controlling for the effects of the other contrasts and the multilevel structure of the data, participants who engaged in intragroup communication while anticipating intergroup contact scored, on average, 0.50 points higher on the 7-point scale measuring stereotype application than participants in the remaining three conditions. As hypothesized, the first control contrast did not significantly affect stereotype application, *p* > .05, but the second control contrast indicated that participants applied more stereotypes to the outgroup after intragroup communication without anticipated face-to-face contact than after individual thought without anticipated face-to-face contact, γ = 0.35 (*SD* = 1.88), *t*(50) = 2.16, *p* = .04. This γ coefficient means that, controlling for the effects of the other contrasts and the multilevel structure of the data, participants who engaged in intragroup communication without anticipating intergroup contact scored, on average, 0.35 points higher on stereotype application than participants in the individual thought without anticipated face-to-face contact condition. And finally, as hypothesized none of the contrasts affected the control measure meta-stereotype application, *p*s > .25.

Thus, anticipating intergroup contact changes intergroup perceptions that can be utilized to buffer against anticipated intergroup hostility only after intragroup interaction. These effects were relatively small yet highly consistent over steeling measures. Besides isolated effects on stereotype application, no such effects emerged on intergroup perceptions that cannot strengthen defensive steeling.

#### Mediation analyses

We hypothesized that hostility anecdotes would mediate the effects of anticipating face-to-face intergroup contact on steeling. To investigate this, we first estimated the effects of anticipated face-to-face contact on the steeling measures within the intragroup communication condition. These analyses were corrected for the different *n*s per cell resulting from the post-hoc design simplification. The effects were again significant for ingroup’s attitude towards the outgroup, *t*(24) = -2.71, *p* = .01, meta-stereotype valence, *t*(24) = 2.69, *p* = .01, and marginally significant for identification, *t*(24) = 1.79, *p* = .09. Subsequently, we estimated the effects of hostility anecdotes (the proposed mediator) on these three steeling variables, while controlling for the effect of anticipating direct intergroup contact (the independent variable). When entered together with hostility anecdotes, the effect of anticipating face-to-face contact on identification was no longer significant, *t*(23) = 0.65, *p* = .52, while the effect of hostility anecdotes was still significant, *t*(23) = 2.46, *p* = .02. There were no significant effects of hostility anecdotes on ingroup’s attitude towards the outgroup or meta-stereotype valence, *p*s > .25. These results suggested a 2-2-1 multilevel mediation from group-level anticipated face-to-face contact, via group-level hostility anecdotes, to individual-level identification. However, they are inconsistent with models assuming that talking about intergroup hostility mediates the relation between anticipated face-to-face contact and ingroup’s attitude towards the outgroup or meta-stereotype valence.

Because Mplus is better equipped to test multilevel mediation, we conducted a 2-2-1 mediation analysis with one-tailed hypothesis tests using multilevel structural equation modelling (MSEM [77]) in Mplus [78] to estimate mediation pattern suggested by the HLM estimations. The indirect effect of anticipated face-to-face contact on identification via hostility anecdotes was marginal, *b* = 0.30, 90% CI [-0.01, 0.60], *p*_one-tailed_ = .05. Following Preacher et al.[77] we report one-tailed MSEM analyses, all other test results are two-tailed. Although this finding should be interpreted with caution because of the small sample size and the marginal significance, it is consistent with the hypothesis that anticipating intergroup contact encourages group members to share anecdotes about experiences with ingroup-directed hostility, which in turn enhances steeling on ingroup identification (see Fig 4). Thus, intragroup communication while anticipating face-to-face intergroup contact apparently facilitates aspects of defensive steeling because this anticipated contact is construed as relatively hostile.

**Fig 4:** Mediation analysis. A multilevel structural equation modelling 2-2-1 mediation analysis with one-tailed hypothesis tests (Preacher et al., 2010) estimated a marginal indirect effect of independent variable (IV) anticipated face-to-face contact on dependent variable (DV) identification via hostility anecdotes, *b* = 0.30, 90% CI [-0.01, 0.60], *p*_one-tailed_ = .05. Although they should be interpreted with caution, depicted estimated coefficients are consistent with a mediational model in which intragroup communication with (versus without) anticipated face-to-face intergroup contact encourages group members to share anecdotes about their personal experiences with ingroup-directed hostility, which in turn enhances ingroup identification.

Because *ingroup’s attitude towards the outgroup*, *meta-stereotype valence*, and *identification* showed similar patterns, we exploratively tested for possible 2-1-1 multilevel mediations with a group-level independent variable (the contrast specified above) in Mplus [78] using the syntax suggested by Preacher et al.[77]. However, no clear evidence of mediation was found, *p*s_one-tailed_ > .05. Thus, there is no consistent evidence that any of the questionnaire variables may have mediated the effects.

## Experiment 2

Experiment 1 showed that intragroup communication while anticipating intergroup contact leads to steeling. The finding that discussing intergroup hostility anecdotes marginally mediated some of these effects suggests that steeling is a defensive reaction to anticipated (somewhat hostile) contact. Sharing such anecdotes presumably raises feelings of discomfort. The interpretation of steeling as a defensive response to reduce the (mild) discomfort posed by imminent intergroup contact seemed supported by null results on most control variables that lacked analogous potential to be used as defensive tools. But better still would be to have measured discomfort and threat in reaction to the intragroup discussions directly. Thus, we conducted a follow-up experiment.

In Experiment 2, new participants (from the same ingroup) listened to the discussions of Experiment 1. Afterwards, they answered questions about the outgroup. The key dependent variables were emotions displaying intergroup discomfort. If steeling is indeed defensive, we hypothesized that discomfort levels should be higher (although possibly still mild) among participants who listened to those group discussions that resulted in steeling. Specifically, we predicted more discomfort among participants who listened to discussions from the anticipated face-to-face contact condition in Experiment 1, compared with participants who listened to discussions from the no anticipation condition. In the current view, individuals need to actively engage in intragroup communication in order to effectively steel themselves against anticipated intergroup hostility. Although listening to audio-recordings of intragroup communication may simulate communication effects to some extent (cf. effects of video-recorded communication [27]), we did not expect adequate levels of steeling in participants who merely listened to intragroup communication. Hence, we expected discomfort among participants who listened to ingroup members collectively anticipating an intergroup confrontation (i.e., those group discussions that resulted in steeling). We measured outgroup-related discomfort as well as actual threat. Because the emotion-evoking potential of outgroups depends on their salient characteristics and the current outgroup was not truly (physically) dangerous, effects might be stronger for the former (cf. [79,80]). Thus, we expected that listening to ingroup members preparing collectively for an intergroup confrontation causes participants to experience discomfort rather than severe threat.

### Method

#### Participants and design

Forty-one students (16 men, age *M* = 22.93, *SD* = 1.94) were randomly assigned to a no anticipation (control) condition or an anticipated face-to-face contact condition.

#### Procedure

The experiment was presented on computers using Qualtrics. After providing informed consent, participants were invited to imagine participating in Experiment 1. To ensure that any effects would be due to differences in communication alone, participants were blind to experimental condition: The procedure made no reference to intergroup contact. There were two conditions: Participants listened to a recording from either the anticipated face-to-face contact condition in Experiment 1 or the no anticipation condition. Within conditions, all Experiment 1 recordings were randomly assigned to participants. Finally, participants filled out an intergroup anxiety measure (including discomfort-related items) and some exploratory measures, demographic and control questions, and were debriefed. The exploratory measures included intergroup conflict intentions, a textual social and a pictorial social distance measure. Because these measures did not show significant effects, the results will not be discussed here but details are available upon request.

#### Measures

An 11-item scale distinguished two intergroup anxiety components: *Discomfort* (“I feel uncomfortable / uneasy in the presence of stadjers”) and *threat* (“I feel threatened / anxious in the presence of stadjers”) on a scale from 1 (*strongly disagree*) to 7 (*strongly agree*). These items were randomly alternated with items for exploratory investigation of anxiety (e.g., “I feel self-conscious / good in the presence of stadjers”).

Control questions measured whether participants were students, whether they had participated in Experiment 1, how strongly they identified with students and with the outgroup, both single-item measures on a scale from 1 (*Absolutely not*) to 7 (*Absolutely*), how well participants heard the audio recording, on a scale from 1 (*The conversation was completely inaudible to me*) to 7 (*The conversation was clearly audible to me*), and how vividly they could imagine being part of the conversation, on a scale from 1 (*It did not feel as if I was one of the students in the conversation at all*) to 7 (*It felt very strongly as if I was one of the students in the conversation*).

### Results

#### Analytic strategy

Several confirmatory factor analyses were conducted in the R package Lavaan (Rosseel, 2012) to investigate whether discomfort and threat constituted two correlated, yet different factors of intergroup anxiety or were better represented as a single measure. Multivariate analyses of variance were used to check comparability of the two conditions and to test the two hypotheses 1) that recordings of ingroup members anticipating intergroup contact would instigate more discomfort than recordings without such anticipation, and 2) that this effect would not occur for intergroup anxiety related threat.

#### Data preparation

Prior to analyses, we removed one participant who indicated that the audio recording was inaudible, leaving 20 participants per condition. All participants confirmed that they were students and that they had not participated in Experiment 1. There were no differences between conditions in identification with students (*M* = 5.20, *SD* = 1.16), *F*(1,38) = 1.20, *p* = .28, η_p_^2^ = .03, or with the outgroup (*M* = 3.05, *SD* = 1.40), *F*(1,38) = 2.62, *p* = .11, η_p_^2^ = .07. Another MANOVA indicated that participants in both conditions heard the conversation on the audio tapes equally well (*M* = 5.10, *SD* = 0.24), *F*(1,38) = 1.09, *p* = .30, η_p_^2^ = .03, and imagined themselves participating in the conversation to a similar extent (*M* = 3.93, *SD* = 0.25), *F*(1,38) = 0.26, *p* = .62, η_p_^2^ = .01.

Mahalanobis distance analyses revealed no multivariate outliers. One univariate outlier on discomfort in the no anticipation condition deviated more than 1.5 interquartile ranges from the condition mean and was removed. The two-factor model representing discomfort and threat as related yet distinct facets of anxiety provided a good fit, *χ* ^2^ (1) = 2.14, *p* = .14, CFI = .99, SRMR = .02. Although these explorative results should be interpreted with caution because of the small sample size, this model fit the data better than the one-factor model, *χ* ^*2*^_*diff*_ = 12.86, *p* < .001.

#### Discomfort and threat

As expected, a MANOVA revealed that participants in the anticipated face-to-face contact condition experienced more (although still mild) discomfort (*M* = 2.90, *SD* = 1.35) than participants in the no anticipation condition (*M* = 2.16, *SD* = 0.78), *F*(1,37) = 4.33, *p* = .04, η_p_^2^ = .11, whereas all participants experienced threat to the same extent (*M* = 2.03, *SD* = 1.06), *F*(1,37) = 0.82, *p* = .37, η_p_^2^ = .02. Thus, listening to ingroup members anticipating face-to-face intergroup contact evoked more discomfort than listening to intragroup conversations without anticipated face-to-face contact. This supported the nature of steeling after intragroup communication as a defensive reaction to prepare for an uncomfortable intergroup confrontation.

## General Discussion

The current experiments investigated the influences of intragroup communication and anticipating intergroup contact on intergroup perceptions and intergroup discomfort. In Experiment 1, content analyses of the discussions revealed that anticipating intergroup contact leads individuals to share more anecdotes about intergroup hostility, rather than to imagine positive intergroup contact. Thus, although experimental work has suggested that individually imagined contact may have some benefits [81] (but see [40]), negative concerns emerged in *spontaneous* intragroup discussions in a contentious context when group members expected to actually meet with the outgroup. Multilevel analyses indicated that intragroup communication—but not individual thought—while anticipating intergroup contact leads to steeling: Participants develop an impression that the outgroup is collectively devalued, they romanticize meta-stereotypes, and identify more strongly with their ingroup. Tentative estimations from mediation analyses were consistent with the assumption that sharing hostility anecdotes boosts individuals’ subsequent ingroup identification. Although this finding should be interpreted with caution because of the small sample size and the marginal significance, it supports the hypothesis that anticipating intergroup contact motivates group members to share anecdotes about experiences with ingroup-directed hostility, which in turn enhances steeling on ingroup identification. Thus, small groups that anticipated face-to-face intergroup contact collectively constructed a shared reality of the outgroup as relatively hostile and—as an apparent, partial consequence—steeled themselves against a negative intergroup confrontation. This finding extends the elaborated social identity model [58] by revealing that individuals may reposition their social identity and corresponding social perceptions in reaction to an outgroup’s *anticipated* reactions to the ingroup, well before actual outgroup behavior takes place.

Of theoretical interest is the finding that steeling only occurred in groups collectively anticipating a real-life discussion with an antagonistic outgroup. Like communication without anticipation of intergroup contact, intragroup communication while anticipating more *indirect* forms of intergroup contact (i.e., sending or mutual exchange of written messages) did not cause group members to steel themselves against an uncomfortable intergroup encounter. The difference between anticipation of dynamic intergroup interaction and more static forms of communication (i.e., mere sending or receiving) complements classical research on communication roles and cognitive tuning. Whereas Zajonc (1960) established that different cognitive structures are activated by communicators who primarily anticipate receiving versus sending information, the present findings indicate that some cognitive changes may only emerge when people anticipate a dynamic succession of sending *and* receiving information.

One explanation for this is that anticipating a real-life intergroup discussion involves anxiety-arousing elements that are not or less present in indirect contact [82,83]. Another explanation involves anonymity. The need for steeling may be stronger when facing real-life contact because written messages may be exchanged anonymously and, hence, arouse less discomfort and threat. Moreover, although previous research suggests that mere outgroup priming may be sufficient to activate intergroup interaction-related behavior [9], Experiment 1 showed that participants only brought up hostility anecdotes if they anticipated an intergroup interaction. This discrepancy may be due to the fact that Cesario and colleagues [9] used subliminal priming of outgroups. Additionally, the emergence of hostile versus benevolent behavior in their studies was moderated by participants’ implicit attitudes towards the outgroup, which were not measured in the current experiment. These speculations remain to be tested empirically. Nonetheless, the current results reveal a consistent pattern of steeling in group members who talked in small groups while anticipating real-life intergroup contact—which is, ironically, the kind of contact in most studies on intergroup contact as an intervention [3].

It is noteworthy that steeling effects were also witnessed in increased ingroup identification. This effect was not found in some previous studies (e.g., [27] Studies 1–3), where participants did *not* anticipate meeting with the outgroup. Additionally, unexpected effects were found on stereotype application. Although we did not conceive of stereotype application as steeling, in some situations stronger application of stereotypic traits may help group members to prepare for an upcoming intergroup interaction. For instance, perception of outgroup members as extremely persistent naggers may have helped Experiment 1 participants to prepare for the worst—a coping strategy that renders harm from disappointment unlikely. Future research could explore this.

Although participants who engaged in intragroup communication while anticipating intergroup contact judged meta-stereotypic traits more positively, they did not perceive the outgroup’s attitude towards the ingroup to be more positive. This pattern is consistent with social creativity, in which group members reject and reverse the negative valence of meta-stereotypes applied to their group [17]. Although Experiment 1 did provide evidence for romanticization of meta-stereotypes, the hypothesized role of meta-stereotype *activation* in anticipating intergroup contact was not supported—possibly due to the method used to gauge activation of meta-stereotypes.

Null findings in Experiment 1 on control variables provide some additional checks on the assumption that the steeling process is mainly focused on rallying the ingroup by rousing the anxieties surrounding the immanent intergroup contact. This interpretation was empirically strengthened by Experiment 2, which revealed that listening to the intragroup discussion from the anticipated face-to-face contact condition of Experiment 1 incited more intergroup anxiety-related emotions (in this intergroup context, discomfort) than the no anticipation condition. This effect emerged even though participants themselves did not anticipate contact. Lee, Gelfand, and Kashima [44] showed that people are more motivated to tell distorted stories about intergroup conflicts in which their friends are involved, for instance by blaming the outgroup and exonerating the ingroup. The current research additionally shows that narratives supporting outgroup blame (i.e., anecdotes about the outgroup’s hostility) may be combined with romanticization rather than denial of blameworthy characteristics. Moreover, both investigations demonstrate the power of intragroup narratives in a relatively neutral and arbitrary laboratory setting—thereby pointing to the potential for truly devastating effects on intergroup conflict escalation in richer and more powerful real-world situations. Taken together, the present research shows that when groups anticipate intergroup contact, the ability to have an ingroup discussion leads to accentuation of uncomfortable thoughts about intergroup contact and consequent steeling against the anticipated intergroup hostility.

At first blush, the transformation of individual group members’ perceptions after intragroup discussion seem consistent with group polarization [84]. For two reasons however, the current results cannot be explained as straightforward polarization effects. One is that we found an effect of intragroup communication *provided that* group members anticipated face-to-face intergroup contact, rather than a main effect of communication. In addition, the romanticization effects were for negative meta-stereotypes to become *less* negative (i.e., a shift more consistent with depolarization). Overall, the steeling effects are reminiscent of the psychological function of groupthink, defined as “mutual enhancement of self-esteem and morale” [70] (p. 88). An imminent confrontation with an antagonistic outgroup requires immediate decisions regarding the course of action, increasing pressure towards consensus and hence facilitating groupthink. Some steeling effects indeed echo aspects of the groupthink processes described by Janis. For instance, romanticization of negative meta-stereotypes may emerge because “victims of groupthink believe unquestioningly in the inherent morality of their ingroup” [70](p. 86). But on balance steeling appears to be something qualitatively different. Janis [70] (p. 86) states that “laughing together about a danger signal, which labels it as a purely laughing matter, is a characteristic manifestation of groupthink.” As this research has shown, steeling centers on the opposite response of defensive toughening up to face the enemy. In other words, the small group discussions in this research had effects that, in many ways, ran opposite to those predicted by groupthink (for similar findings see [85,86]).

These findings are more consistent with saying-is-believing effects. That is, sharing hostility anecdotes increased group members’ belief in outgroup hostility, which led them to steel themselves. Moreover, when anticipating an intergroup discussion, group members may plan to resist the uncomfortable experience of unilateral condemnation by the outgroup by intending to communicate certain messages rather than others. For instance, they may plan to express their appreciation of meta-stereotypic traits and to stress that the ingroup is not that fond of the outgroup either. Such intentions of what group members plan to say also influence their perceptions [87]. Thus, the tone and content of anticipated intergroup communication may play a role in the manifestation of steeling in individuals’ intergroup perceptions. Steeling seems an additive effect of what is actually said in intragroup conversations (i.e., hostility anecdotes) and what group members plan to say during intergroup contact. Future research may disentangle these two influences.

The fact that intragroup communication in anticipation of intergroup contact led to more negative intergroup perceptions of the outgroup suggests that ingroup norms may have changed as a result of the discussion. More particularly, the perception of what the ingroup believes about the outgroup is essentially a descriptive norm: “We do not like them”[36] (cf. [27]). This is also revealed in the content analysis, where anticipated face-to-face contact sparked the sharing of anecdotes about personal experiences with (mild) outgroup hostility. Just as observation of positive intergroup contact can improve intergroup relations by validating a positive social or shared reality (cf. [22,23,88]) and providing a positive group norm [31,37,38], anecdotes describing negative intergroup contact may deteriorate intergroup relations by negative norm setting. Extended contact (i.e., learning about others’ positive intergroup contact) improves intergroup relations by amongst other processes reducing intergroup anxiety [35]. Experiment 2 suggested its negative counterpart: Intragroup communications among those who anticipated face-to-face intergroup contact with a hostile outgroup *increased* (mild) intergroup discomfort among an ingroup audience who were unaware of that contact was imminent.

Together, the findings from Experiments 1 and 2 findings open interesting venues for future research. For example, the impact of a mental representation (such as a particularly hostile outgroup) on perceptions and behavior depends on its motivational relevance [89]. Several previous studies have demonstrated that goal fulfillment decreases the accessibility of related constructs [90,91]. In the current research, steeling apparently served the goal to adequately prepare for an uncomfortable confrontation with an antagonistic outgroup. This implies that group members who effectively steeled themselves against anticipated hostility should experience reduced intergroup anxiety. Indeed after successful steeling or after successfully withstanding an outgroup’s insults and accusations, promotion-focused group members might even inhibit the mental representation of the outgroup as potentially threatening in order to free cognitive resources for performing the next task (cf. [91]). Future research could explore these issues.

One possible limitation of the current manipulations is that participants may have construed the anticipated face-to-face intergroup contact differently across conditions. People who prepare individually for a discussion with ingroup and outgroup members may be preoccupied with how ingroup members expect them to behave, whereas individuals who prepare for intergroup contact during intragroup communication might instead discuss what “they” will do and how “we” should react. Consequently, the former may construe the anticipated interaction as less intergroup, which leads them to experience less intergroup discomfort or threat and, hence, refrain from steeling themselves. Although this would be consistent with our explanation, we did not measure participants’ construal of the anticipated discussion and so we cannot be entirely certain this was the case. Future research should address this.

To conclude, this research provides new insights into how intergroup perceptions change during intragroup communication. The findings extend the existing intergroup conflict literature, which primarily focuses on intra-individual and intergroup processes. *Intragroup* processes are also pivotal because they shape individual perceptions (cf. [21,23,88]) and set the stage for intergroup behavior [26]. Spontaneous intragroup communication when anticipating intergroup contact evokes (mild) intergroup discomfort and may lead people to subsequently steel themselves against anticipated hostility rather than to open their minds and hearts for constructive intergroup contact. Thus, intragroup processes may partially explain why groups can experience severe conflict even when they never meet.

## Supporting Information

S1 Dataset (SAV)

S2 Dataset (SAV)
